The article "Fine Complex Geological Structure Interpretation Based on Multiscale Seismic Dip Constraint" was published in 2022. Journal: Comput Intell Neurosci.

# Fine Complex Geological Structure Interpretation Based on Multiscale Seismic Dip Constraint

**DOI:** 10.1155/2022/1529935

**Published:** 2022-02-24

**Authors:** Zhenhua Zhang, Zhenan Yao, Pan Wang

**Affiliations:** ^1^College of Geoscience and Surveying Engineering, China University of Mining and Technology (Beijing), Beijing 100083, China; ^2^Engineering Research Center for Seismic Disaster Prevention and Engineering Geological Disaster Detection of Jiangxi Province (East China University of Technology), NanChang, Jiangxi 330013, China; ^3^State Key Laboratory of Nuclear Resources and Environment, East China University of Technology, Nanchang 330013, Jiangxi, China

## Abstract

With the development of seismic exploration technology, geological structure interpretation has become more and more refined, whereas random noise interference, subsalt weak seismic reflection signals, and other issues are also gradually emerged at the same time, which resulted in traditional geological structure interpretation accuracy reduction only relying on single seismic data. A novel technical process integrated time-frequency decomposition of seismic data, seismic dip constraints, and geological structure interpretation is proposed in this paper which is named multiscale seismic dip constraint geological structure interpretation. The technical process contains five steps which first use the basis tracking spectrum decomposition technology to convert the seismic data into the time-frequency domain and then decompose the raw seismic data into coarse scale, fine scale, and deliberate scale through window and threshold methods. Subsequently, execute local layer dip calculation with Hilbert transform and geological structure interpretation on seismic data of different scale, respectively. At last, perform geological structure attribute fusion to obtain fine geological structure interpretation. Synthetic data test and field data test show that through multiscale time-frequency decomposition, high-frequency noise interference can be removed and the subsalt seismic weak signal can be enhanced, and then, high-precision fine complex geological structure interpretation can be obtained with seismic dip constraint. Therefore, the technical process proposed in this paper is effective and can be widely applied in the interpretation of field seismic data.

## 1. Introduction

With the deepening of oil and gas exploration and development, exploration targets are gradually transitioning to deep, small structures, and lithological oil and gas reservoirs, which put forward higher and higher requirements for fine seismic data interpretation technology. Traditional geological structure interpretation is often based on a single seismic section to trace the seismic event to outline the shape of the underground geological structure, which can only be used to explain large geological structures such as obvious stratum boundaries or larger faults. As the depth of the formation increases, the effective geological structure information in the seismic data is often submerged in random noise. At the same time, as the geological age increases, some igneous and gypsum rock formations develop, which will cause the seismic reflection energy of the subsalt formation to weaken. Therefore, it has become an important development trend to make full use of seismic, geological, well logging, and other data to dig out more effective information to complete fine structure interpretation.

In order to make full use of seismic data, geophysicists consider transforming seismic data into frequency domain for analysis to extract more characteristic information. Among them, spectrum decomposition technology is a widely used tool [1]. Time-frequency decomposition technology can be used to describe the nonstationary relationship between time and instantaneous frequency [2]. In the past few decades, it has gradually developed into a powerful tool for seismic signal processing and interpretation [3, 4]. It is widely used in seismic thin layer thickness analysis and hidden low-frequency gas shadow detection and other aspects [5–7]. The classic short-time Fourier transform (STFT) has an inherent window effect [8], so wavelet-based spectrum decomposition method is widely used [9]; this type of method has shown good performance in describing the microstructure and reservoir characteristics, such as continuous wavelet transform [10] and matching pursuit technology [11–13]. Liu and Fomel [14] developed a S transform method based on local attributes [15]; the high resolution spectral decomposition through regularized nonstationary regression was widely used to seismic surface wave suppression and seismic denoising [16, 17]. In recent years, time-frequency decomposition techniques based on the combination of algorithms and inversion schemes have shown greater improvement in time-frequency resolution [18, 19] and time-variant wavelet extraction [20, 21], which makes seismic interpretation more accurate.

As we all know, the stratum dip is an important geological feature, we can use seismic dip to determine structural trends and achieve structure protection. In order to obtain the stratum dip in seismic section, several methods have been proposed, such as local slant stack [22] and plane-wave destruction (PWD) filter [23]. Schleicher et al. [24] compared different methods of local dip computations. In the field of seismic exploration, seismic dip information is often used to seismic data denoising, for example, Lu and Lu [25] constructed structure-oriented filters to suppress random seismic noise. Liu et al. [26] used polynomial fitting and shaping regularization to form a novel seismic noise attenuation method which realized edge-preserving.

Oriented random noise interference, subsalt weak seismic reflection signals, and other issues that reduce the accuracy of geological structure interpretation, and a novel technical process integrated time-frequency decomposition of seismic data, seismic dip constraints, and geological structure interpretation are proposed in this paper which achieved fine geological structure interpretation accurately and efficiently.

## 2. Theory

### 2.1. Time-Frequency Multiscale Decomposition Based on Basis Pursuit

As an important tool for geological structure interpretation, seismic data characteristics are extensively studied, in which spectrum decomposition has been widely used in recent years. Two-dimensional seismic data are composed of multiple seismic records and a seismic record can be expressed as the convolution of seismic wavelet and reflection coefficient sequence. Based on basis pursuit theory, seismic record *s*(*t*) is expressed as a convolution of basis functions *ψ*(*t*, *n*) and coefficient sequences *a*(*t*, *n*):

(1) $$\begin{array}{c} s\left(t\right)=\sum_{n=1}^{N}\left[\psi \left(t,n\right)*a\left(t,n\right)\right], \end{array}$$

where *N* is the number of basis functions, *t* is time, and *n* is the scale parameter that controls the frequency characteristics of the basis functions. Using matrix notation, the equation can be rewritten as

(2) $$\begin{array}{c} s=\left(\begin{array}{ccc} \Psi_{1} & \Psi_{2}. & \Psi_{N} \end{array}\right)\left(\begin{array}{c} a_{1}\\ a_{2}\\ \vdots \\ a_{N} \end{array}\right)+\eta =\mathrm{Da}+\mathrm{\eta ,} \end{array}$$

where **s** is the vector notation of seismic trace *s*(*t*), Ψ_**n**_ is the convolution matrix of basis function *ψ*(*t*, *n*), **a**_**n**_ is the coefficient vector corresponding to Ψ_**n**_, **D** is the waveform dictionary, **a** is the column vector formed by **a**_**n**_, that is a column vector formed by all coefficients *a*(*t*, *n*) arranged in columns, and *η* is random noise. Then, the spectral decomposition result is the distribution of the weight coefficient *a*(*t*, *n*) of the seismic trace mapping in the waveform dictionary **D** in the time-frequency space. The solution of the above equation is a typical basis tracking denoising problem, so based on the solution of the following objective function equation to obtain time-frequency multiscale decomposition,

(3) $$\begin{array}{c} J=\text{min}\left[\frac{1}{2}{\left\|s-Da\right\|}_{2}^{2}+\lambda {\left\|a\right\|}_{1}\right], \end{array}$$

where ‖*∗*‖_1_ represents the *l*_1_ norm, ‖*∗*‖_2_ represents the *l*_2_ norm, and the first term of the objective function *J* represents the data error term based on the *l*_2_ norm, that is, the least square error between the seismic trace and the reconstructed data, and the cost function is *J*. The second term is the *l*_1_ norm constrained regularization term, and *λ* is the trade-off factor, which controls the relative strength of data error and solution sparsity.

### 2.2. Local Layer Dip Calculation with Hilbert Transform

Seismic data are a function of time and space. In the two-dimensional case, the seismic wavefield data are recorded as *P*(*x*, *t*), following the local plane-wave equation as

(4) $$\begin{array}{c} \frac{\partial P\left(x,t\right)}{\partial x}+\sigma \left(x,t\right)\frac{\partial P\left(x,t\right)}{\partial t}=0, \end{array}$$

where *σ*(*x*, *t*) represents local layer dip of seismic data, so

(5) $$\begin{array}{c} \sigma \left(x,t\right)=\frac{-\partial P\left(x,t\right)/\partial x}{\partial P\left(x,t\right)/\partial t}. \end{array}$$

In practical application, the calculation of local layer dip of seismic data *σ*(*x*, *t*) should ignore partial and temporal sampling interval; therefore, *σ*(*x*, *t*) becomes dimensionless defined as

(6) $$\begin{array}{c} \sigma =-\left(\frac{-\partial P\left(x,t\right)/\partial x}{\partial P\left(x,t\right)/\partial t}\right)\cdot \frac{\Delta x}{\Delta t}=-\frac{\partial P/\partial x}{\partial P/\partial y}, \end{array}$$

where Δ*x* and Δ*t* represent time and space sampling interval. As the direct calculation of derivative in the above equation would enhance the high-frequency random noise, Hilbert transform is introduced to redefine the local layer dip as

(7) $$\begin{array}{c} \sigma =-\left(\frac{\partial P/\partial x}{\partial P/\partial y}\right)=-\frac{\mathrm{FF}T^{-1}\left[\tilde{P}\left(x\right)\right]}{\mathrm{FF}T^{-1}\left[\tilde{P}\left(t\right)\right]}=-\frac{\mathrm{FF}T^{-1}\left[1/\sqrt{c_{x}}\tilde{P}\left(x\right)\right]}{\mathrm{FF}T^{-1}\left[1/\sqrt{c_{t}}\tilde{P}\left(t\right)\right]}\approx -\frac{\mathrm{FF}T^{-1}\left[H_{HT}\left(x\right)\right]}{\mathrm{FF}T^{-1}\left[H_{HT}\left(t\right)\right]}\approx -\frac{H_{HTx}}{H_{HTt}}, \end{array}$$

where $\tilde{P}\left(x\right)$ and $\tilde{P}\left(y\right)$ represent the frequency response of the derivative in the *x* and *t* directions, respectively, *c*_*x*_ and *c*_*t*_ are transformation parameters because the local layer dip is dimensionless, so take *c*_*x*_=*c*_*t*_ here, and *H*_*HTx*_ and *H*_*HTy*_ represent the frequency response function of the Hilbert transform along *x* and *t* directions, respectively. With equation (7), the local layer dip of seismic data could be calculated using 2D Hilbert transform instead of directly computing the derivative. In order to avoid the denominator which becomes zero which results in instability, a nonzero constant *ε* is introduced, and the local layer dip calculation expression becomes

(8) $$\begin{array}{c} \sigma \approx -\frac{H_{HTx}}{H_{HTy}+\varepsilon }. \end{array}$$

### 2.3. Multiscale Seismic Dip Constraint Geological Structure Interpretation

In traditional seismic section interpretation, only a single seismic data is used, and lots of effective information is submerged, which reduces the accuracy of geological structure interpretation. At the same time, in the case of strong noise or strong reflective layer shielding, fine geological structure interpretation cannot be realized, and only rely on single scale seismic data. With time-frequency multiscale decomposition and local layer dip calculation technology, a flowchart of multiscale seismic dip constraint geological structure interpretation is proposed, as shown in Figure 1. The whole process can be divided into the following five steps.

- Input the raw seismic data, and use the basis tracking spectrum decomposition technology to convert the seismic data into the time-frequency domain
- Use window and threshold methods to divide seismic data into three scales in the time-frequency domain; three scales are coarse scale, fine scale, and deliberate scale, respectively
- Convert the processed three-scale time-frequency domain data to the time-space domain based on inverse transform
- Execute local layer dip calculation with Hilbert transform and geological structure interpretation on seismic data of different scales, respectively
- By orienting to seismic data of different scales, perform geological structure attribute fusion to obtain fine geological structure interpretation at last

## 3. Synthetic Data Test

A model data is built by convolution of Ricker wavelet and reflection coefficient sequence, as shown in Figure 2(a), in which tilted layer, fault, syncline, and anticline geological structure are included. Because of random noise pollution and little fault displacement, it is easy to dislocate during fault geological interpretation. With multiscale seismic dip constraint geological structure interpretation proposed in this paper, this problem can be easily solved and the accuracy of fault interpretation can be improved. Figures 2(b) and 2(c) show the fine scale and deliberate scale seismic data, respectively, in which the fine scale seismic data contain most of the valid information, and the deliberate scale seismic data are almost all random noise, so geological structure interpretation can be equivalently executed only on fine scale seismic data with deliberate scale seismic data which are abandoned. As shown in Figure 2(d), the local layer dip was calculated, which controls the trend of the event, and the fault can be clearly identified. Therefore, the flowchart of multiscale seismic dip constraint geological structure interpretation stated in this paper is effective.

## 4. Field Data Test

In order to verify the effect of the technique process proposed in this paper, a field pre-stack time migration seismic section was introduced from a working area of Xinjiang Province, China. In the work area, the geological structure is very complex, and a layer of gypsum rock is developed in the Cambrian strata, which leads to weak seismic signal energy in the subsalt strata, as shown in Figure 3. Therefore, it is difficult to identify the subsalt formation and its geological structure on a single seismic profile, which means that the traditional methods are ineffective. Using the technical process proposed in this paper, the local seismic dip and partial geological structure interpretation is accomplished, as shown in Figure 4, in which the subsalt strata and geological structures are clearly displayed as indicated by the red ellipse, and the extension of deep strata is also reflected; it has a great significance for enhancing the continuity of geological structure and stratigraphy. The amplification of the elliptic marking area in Figures 3 and 4 are shown in Figure 5, in which fault structures and stratigraphic structures are clearly presented in seismic dip section copaired with seismic section.

## 5. Conclusions

Due to interferences such as random noise and high-speed salt shielding, it is often impossible to complete accurate geological structure interpretation only relying on a single seismic data. A multiscale seismic dip constraint geological structure interpretation technical process is proposed in this paper, which contains five steps to decompose the raw seismic data into different scales for geological structure interpretation, and then, the interpretation results of various scales of geological structure attributes are combined. Based on synthetic data test and field data test, it shown that high-frequency noise interference can be removed and the subsalt seismic weak signal can be enhanced with multiscale time-frequency decomposition, and fine geological structure interpretation can be obtained using local layer dip calculation, so the multiscale seismic dip constraint geological structure interpretation technical process proposed in this paper is proved effective. In addition, in recent years, oil and gas exploration and development have continued to expand into deep formations, and effective seismic signals have become weak or submerged in random noise. Considering the multiscale decomposition of seismic sections for geological structure interpretation will receive more and more attention.

## Figures and Tables

**Figure 1:** Flowchart of multiscale seismic dip constraint geological structure interpretation.

**Figure 2:** Flowchart of multiscale seismic dip constraint geological structure interpretation. (a) Synthetic seismic data with noise; (b) the fine scale seismic data; (c) the deliberate scale seismic data; (d) local seismic dip.

**Figure 3:** A field pre-stack time migration seismic section.

**Figure 4:** Local seismic dip and partial geological structure interpretation.

**Figure 5:** Amplification show of elliptic marking area in Figures 3 and 4.

## Data Availability

The data used to support the findings of the study are available from the corresponding author upon request.
